The article "High Expression of RIOK2 and NOB1 Predict Human Non-small Cell Lung Cancer Outcomes" was retracted in 2023. Reasons: duplicated images; original data or images not available; unreliable results or conclusions; concerns about the data.

# High Expression of RIOK2 and NOB1 Predict Human Non-small Cell Lung Cancer Outcomes

**DOI:** 10.1038/srep28666

**Published:** 2016-06-27

**Authors:** Kun Liu, Hong-Lin Chen, Shuo Wang, Ming-Ming Gu, Xin-Ming Chen, Shuang-Long Zhang, Kang-Jun Yu, Qing-Sheng You

**Affiliations:** 1 Department of Cardiothoracic Surgery, Affiliated Hospital of Nantong University, Nantong 226001, China; 2 Nantong University, Nantong, 226001, China

## Abstract

Non-small cell lung cancer (NSCLC) is the leading cause of cancer-related mortality worldwide. However, there is a shortage of suitable diagnostic markers for early stages of NSCLC, and therapeutic targets are limited. Right open reading frame (Rio) kinase 2 (RIOK2) and Nin one binding (NOB1) protein are important accessory factors in ribosome assembly and are highly expressed in malignant tumours; moreover, they interact with each other. However, the RIOK2 expression profile and its clinical significance as well as NOB1’s mechanism in NSCLC remain unknown. In this study, NSCLC cell lines and 15 NSCLC tumour tissues (paired with adjacent normal lung tissues) were collected for a real-time quantitative PCR (RT-qPCR) analysis. In addition, 153 NSCLC cases and 27 normal lung tissues were used in an immunohistochemical analysis to evaluate the RIOK2 and NOB1 expression profiles, their clinicopathological factors in NSCLC and their correlations with prognoses. RIOK2 and NOB1 were highly expressed in NSCLC cells and tissues, and their expression profiles were significantly associated with the Tumour Node Metastasis (TNM) clinical stage, lymph node metastasis, and differentiation. RIOK2 expression was correlated with NOB1. The results suggested that simultaneously determining the expression of RIOK2 and NOB1 will improve the diagnostic rate in early stages of NSCLC. Moreover, RIOK2 and NOB1 might be potential targets for NSCLC therapy.

Lung cancer is the most common global cancer and the second leading cause of cancer death. Non-small cell lung cancer (NSCLC) is the most common lung cancer type, accounting for approximately 85 to 90% of lung cancers^1^. Surgical resection has been the single most consistent and successful method for treatment of early-stage lung cancer^2^,^3^. However, prognoses are still poor after surgical resection, and the 5-year survival rate is very low^4^. Thus, it is important to predict the prognosis for resected NSCLC.

The nin one binding (NOB1) protein has recently been found to be highly expressed in several cancers, and it also plays a significant role in tumourigenesis. It is related to cancer prognosis^5^, such as for thyroid carcinoma^6^, ovarian cancer^7^, chronic myeloid leukaemia^8^, glioma^9^ and spleen cancer^10^. The NOB1 protein is a subunit of the 26S proteasome, which plays a crucial role in protease functions and RNA metabolism^11^. Our previous studies have shown that abnormal NOB1 expression is related to lung cancer, especially NSCLC; moreover, NOB1 is significantly highly expressed in NSCLC patients, and this expression is associated with the TNM stage, lymph node metastasis and histopathological grade^12^,^13^. However, the underlying mechanism is unknown.

The article "High Expression of RIOK2 and NOB1 Predict Human Non-small Cell Lung Cancer Outcomes" was retracted in 2023. Reasons: duplicated images; original data or images not available; unreliable results or conclusions; concerns about the data.

Right open reading frame (RIO) kinase 2 (RIOK2) is a member of the RIO family^14^. RIOK1 (or RIOK2) plays key roles in synthesis of the 40S ribosomal subunit by promoting 20S pre-rRNA transfer to mature 18S rRNA^15^,^16^,^17^,^18^. An *in vitro* binding assay has confirmed that RIOK2 directly binds ribosomal proteins Rps15, Rps14 and Rps5 and directly or indirectly interacts with many ribosomal components (e.g., NOB1). In addition, NOB1 interacts with the ribosomal proteins Rps5 and Rps14, and GST pulldown assays have confirmed that RIOK2 interacts with NOB1^19^. Moreover, RIO molecules are highly expressed in many tumours^20^,^21^,^22^,^23^,^24^; however, previous studies have not evaluated the relationship between RIOK2 and NSCLC.

In this study, we investigated the expression of both RIOK2 and NOB1 in the same NSCLC patients. We further assessed the clinicopathological significance of RIOK2 and NOB1 and the prognostic value of the relationship between these proteins.

## Materials and Methods

### NSCLC cell lines and cell culture

NSCLC cell lines (A549, H1299, H1975 and H1650) and the human lung cell line BEAS-2B were obtained from the cell bank of the Central South University in Changsha, China. These cells were cultured in Dulbecco’s modified Eagle’s medium (DMEM) (Gibco, USA) with 10% foetal bovine serum (FBS) (Gibco, USA) at 37 °C in a 5% CO_2_ incubator.

### Patient specimens

NSCLC tumour tissues and paired adjacent normal lung tissues were obtained from 15 patients who had undergone primary surgical NSCLC resection at the Affiliated Hospital of Nantong University, and the tissues were fresh frozen. In addition, 153 cases of formalin-fixed and paraffin-embedded NSCLC tumour tissues and 27 normal lung tissues were collected from the Department of Pathology of the Affiliated Hospital of Nantong University from 2005 to 2011. None of the patients had received preoperative chemotherapy or radiotherapy prior to surgery. The recorded clinical data and diagnoses of all tissues were confirmed by two independent pathologists. The histological grades and clinical stages of all of the NSCLC patients were evaluated according to the pathological results after surgery.

The article "High Expression of RIOK2 and NOB1 Predict Human Non-small Cell Lung Cancer Outcomes" was retracted in 2023. Reasons: duplicated images; original data or images not available; unreliable results or conclusions; concerns about the data.

The clinical data of 153 NSCLC patients included the following: gender (male, n = 82, female, n = 71), age (<60 years, n = 71; ≥60 years, n = 82), tumour diameter (<3 cm, n = 94; ≥3, n = 59), TNM clinical stage (stages I and II, n = 103; stage III, n = 50), lymph node metastasis (No, n = 63; Yes, n = 90) and differentiation (well, n = 2; moderately, n = 99; and poorly, n = 52). In addition, 15 NSCLC tumour tissues and paired adjacent normal lung tissues were collected for reverse-transcriptase quantitative polymerase chain reaction (RT-qPCR) analysis. All of the patients provided written informed consent before participation in this study. The study protocol was approved by the Human Research Ethics Committee of the Affiliated Hospital of Nantong University, and all of the experiments were performed in accordance with the approved guidelines of the Affiliated Hospital of Nantong University.

### RT-qPCR

Total RNA from the cell lines and frozen tissues described above was extracted using TRIzol^®^ Reagent (Thermo Fisher Scientific, USA) according to the manufacturer’s instructions. The RIOK2 and NOB1 mRNA levels were detected with a one-step RT-qPCR reaction using a SuperScript^®^ III Platinum^®^ SYBR^®^ Green One-Step qRT-PCR Kit (Thermo Fisher Scientific, USA) according to the manufacturer’s instructions. The PCR primer sequences for RIOK2 and NOB1 were designed as follows: RIOK2, forward 5′-ACAACAGGCAAGATGGTCA-3′ and reverse 5′-GACGACAAGGCAATTAGATGAG-3′; NOB1, forward 5′-ACATACCAGTTGGAAGCAGAG-3′ and reverse 5′-CAGGTTCTCAGGCTCACAAG-3′. GAPDH was used as an internal control, and the primers were as follows: forward 5′-GAAGGTGAAGGTCGGAGTC-3′ and reverse 5′-GAAGATGGTGATGGGATTTC-3′. The RT-qPCR reaction conditions included reverse transcription at 50 °C for 3 min and then preheating at 95 °C for 5 min, which was followed by 45 cycles of denaturation at 95 °C for 15 sec, annealing at 60 °C for 30 sec, and extension at 72 °C for 30 sec. The RIOK2 and NOB1 mRNA levels were normalized to that of GAPDH. The experiment was performed in triplicate, and the results were analysed with the 2^−ΔΔCt^ method^25^.

### Immunohistochemistry

Immunohistochemistry (IHC) staining was performed using an Envision Plus/Horseradish Peroxidase system (DAKO, USA), and 4 μm sections were dewaxed and rehydrated through descending grades of alcohol to distilled water and then incubated in 0.3% hydrogen peroxide and absolute methanol to block endogenous peroxidase activity. Subsequently, the sections were pressure cooked in sodium citrate buffer (10 mM sodium-citrate monohydrate, pH 6.0) for antigen retrieval. The sections were then incubated with rabbit anti-RIOK2 polyclonal antibody (Abcam, USA, dilution 1:100) and rabbit anti-NOB1 polyclonal antibody (Abcam, USA, dilution 1:100) overnight at 4 °C. After being washed with PBS, the slides was incubated with the Envision Plus secondary antibody for 30 min and then with diaminobenzidine for 5 min. Appropriate positive and negative controls (incubation with secondary antibody alone) were stained in parallel.

The article "High Expression of RIOK2 and NOB1 Predict Human Non-small Cell Lung Cancer Outcomes" was retracted in 2023. Reasons: duplicated images; original data or images not available; unreliable results or conclusions; concerns about the data.

The percentages of RIOK2 and NOB1 positive cells were scored in four categories according to staining as follows: 0 for 0%, 1 for 1–33%, 2 for 34–66%, and 3 for 67–100%. The sum of the percentages and intensity scores was used as the final staining score as follows: 0 for-(no staining), 1–3 for + (weak staining), 4–6 for ++ (moderate staining), and 7–9 for +++ (intense staining).

### Western blot

The tissue samples were homogenized in T-PER^®^ Tissue Protein Extraction Reagent (Thermo Fisher Scientific, USA) and centrifuged at 10,000 g for 5 min to pellet the tissue debris. The supernatant was then collected, and the total protein was separated by sodium dodecyl sulphate-polyacrylamide gel electrophoresis (SDS-PAGE), electroblotted onto polyvinylidene difluoride filter (PVDF) membranes (Millipore, USA), and then blocked with 5% skim milk in TBST (20 mM Tris, 150 mM NaCl, 0.05% Tween-20, pH 7.5) buffer for 2 h at room temperature. Subsequently, the membranes were incubated with rabbit anti-RIOK2 polyclonal antibody (Abcam, USA; 1:100 dilution) or mouse-anti-human β-actin antibody (Abcam, USA; 1:500 dilution) as an internal control. Then, the membranes were washed in TBST and incubated with a goat anti-rabbit or goat anti-mouse HRP-conjugated secondary antibody (Abcam, USA; 1:1000 dilution) at room temperature for 2 h. Finally, the specific proteins were detected with a Novex^®^ ECL Chemiluminescent Substrate Reagent Kit (Thermo Fisher Scientific, USA), and the membranes were exposed to films (Kodak, USA).

### Statistical analysis

All of the data were analysed using SPSS 19.0 statistics software (SPSS, USA) and STATA 12.0 (Stata, USA). The statistical analysis of RT-qPCR data was performed using the *t*-test for comparisons between two groups. The Pearson *χ*2 test and Fisher’s exact test were used to analyse the associations between RIOK2 or NOB1 expression and the clinicopathological parameters. The survival curves were analysed using the Kaplan-Meier method and log-rank test. Prognostic factor significance in the univariate models was evaluated with a multivariate Cox proportional hazard model. For all of the analyses, *P* < 0.05 was considered to be statistically significant.

## Results

### RIOK2 and NOB1 mRNA expression levels in the NSCLC cell lines and tissues

The RIOK2 and NOB1 mRNA levels in the NSCLC cells (A549, H1299, H1975 and H1650) and normal human lung cells (BEAS-2B) were determined by RT-qPCR. Compared with the BEAS-2B cells, the relative mRNA levels of RIOK2 and NOB1 in the NSCLC cell lines were all highly expressed (Fig. 1).

The article "High Expression of RIOK2 and NOB1 Predict Human Non-small Cell Lung Cancer Outcomes" was retracted in 2023. Reasons: duplicated images; original data or images not available; unreliable results or conclusions; concerns about the data.

The NSCLC tumour and paired adjacent normal lung tissues from 15 patients were also used to evaluate the RIOK2 and NOB1 mRNA levels by RT-qPCR. As shown in Fig. 2, the mean values of RIOK2 mRNA in the tumour and normal tissues were 2.16 ± 0.57 and 0.46 ± 0.21, respectively. The mRNA expression of RIOK2 in the NSCLC tumour tissues was significantly higher than that in the normal lung tissues (*P* < 0.001). In addition, the mean levels of NOB1 mRNA in the tumour and normal tissues were 1.06 ± 0.23 and 0.87 ± 0.16, respectively. The NOB1 mRNA level in the NSCLC tumour tissues was significantly higher than that in the normal lung tissues (*P* = 0.014).

### Expression profiles of RIOK2 and NOB1 in the NSCLC patients analysed by IHC

A IHC analysis with TMA was performed to confirm the RIOK2 and NOB1 expression levels in the 153 NSCLC patients (compared with 27 case normal lung tissue patients). The RIOK2 expression was significantly upregulated in the NSCLC patients and absent or low in the normal lung tissues, and high RIOK2 expression levels were observed in the NSCLC patients by western blot assays of the fresh-frozen tissues (Fig. 3). RIOK2 and NOB1 both presented positive staining in the cytoplasm of tumour cells. High RIOK2 expression was observed in 45.75% (70/153) of tumours compared with 7.41% (2/27) of normal tissues, and this difference was statistically significant (χ^2^ = 20.204, *P* < 0.001). Overexpression of NOB1 was observed in 43.14% (66/153) of tumours compared with 3.70% (1/27) of normal tissues, and this difference was statistically significant (χ^2^ = 25.954, *P* < 0.001).

### Association of RIOK2 and/or NOB1 expression with clinicopathological parameters in NSCLC patients

The association of RIOK2 or NOB1 expression with clinicopathological parameters is shown in Table 1. Significant associations were observed between the positive expression of RIOK2 and the TNM clinical stage (*P* < 0.001), lymph node metastasis (*P* < 0.001), and differentiation (*P* = 0.018). In addition, the positive expression of NOB1 protein was also associated with the TNM clinical stage (*P* = 0.003), lymph node metastasis (*P* = 0.017), and differentiation (*P* = 0.030). However, RIOK2 and NOB1 expression levels were not significantly associated with gender, age, smoking status, or tumour diameter (all *P* > 0.05).

Furthermore, a Pearson’s correlation analysis was performed, and the results showed a significant positive correlation between the expression of RIOK2 and NOB1 in 153 cases of NSCLC (χ^2^ = 0.606, *P* < 0.001) as shown in Fig. 4.

The article "High Expression of RIOK2 and NOB1 Predict Human Non-small Cell Lung Cancer Outcomes" was retracted in 2023. Reasons: duplicated images; original data or images not available; unreliable results or conclusions; concerns about the data.

### Prognostic value of RIOK2 or NOB1 expression in NSCLC patients

A multivariate analysis was performed using the Cox proportional hazards model for all of the significant variables in the univariate analysis. In the univariate survival analysis, high RIOK2 expression (HR = 2.878; *P* < 0.001), high NOB1 expression (HR = 2.030; *P* = 0.001), tumour diameter (HR = 1.641, *P* = 0.021), TNM clinical stage (HR = 3.381; *P* < 0.001), lymph node metastasis (HR = 1.795; *P* = 0.010) and differentiation (HR = 2.172; *P* < 0.001) were associated with the overall survival rate (Table 2). The significance of these prognostic factors in the univariate models was evaluated in a multivariate Cox regression model, and the results demonstrated that RIOK2 overexpression (HR = 2.105; *P* = 0.003), NOB1 overexpression (HR = 1.858; *P* = 0.005) and TNM clinical stage (HR = 2.166; *P* < 0.002) were independent prognostic factors for poor outcomes (Table 2). As shown in the Kaplan–Meier survival curves (Fig. 5), NSCLC patients who presented with high RIOK2 or NOB1 expression had poor overall survival rates compared with patients who presented with low expression (RIOK2: *P* < 0.001; NOB1: *P* = 0.001), and patients who presented with high expression levels of both RIOK2 and NOB1 had poorer overall survival rates compared with patients who presented with low expression levels of RIOK2 or NOB1 (*P* < 0.001).

## Discussion

Lung cancer, especially NSCLC, is a malignant tumour with high mortality^1^,^2^,^3^. Thus, it is extremely urgent and important to clarify the pathogenesis of NSCLC and identify potential therapeutic targets.

The RIO family of proteins includes RIOK1, RIOK2 and RIOK3, which have the characteristics of kinases but lack a typical kinase domain; therefore, they are referred to as atypical kinases^14^. RIOK1 and RIOK2 are highly conserved in eukaryotes including yeast and mammals, and RIOK3 is expressed in only eukaryotic cells^14^,^26^. RIOKs are highly expressed in head-and-neck carcinoma^20^, glioblastoma^21^, colon cancer^22^, pancreatic cancer^23^, and melanoma^24^. RIOK1 and RIOK2 are overexpressed in glioblastoma cells in an Akt-dependent manner, and down-regulated expression of RIOK1 or RIOK2 disrupts Akt signalling and causes cell cycle exit, apoptosis, and chemosensitivity in glioblastoma cells by inducing p53 activity^27^. RIOK proteins can also regulate the ERK, Ras, NFκB and Hedgehog pathways^28^,^29^,^30^,^31^,^32^, and they are the target genes of the oncogene *myc*^33^. However, except in glioblastoma, the mechanism of RIOK in other tumours has been unknown until now. In this study, RIOK2 was detected in NSCLC cell lines and tissues from NSCLC patients. RIOK2 was highly expressed in the NSCLC cell lines and tissues compared with the normal cell and tissues (Figs 1 and 2). The results of the IHC analysis showed that the positive expression of RIOK2 was significantly associated with the TNM clinical stage (*P* < 0.001), lymph node metastasis (*P* < 0.001), and differentiation (*P* = 0.018) (Fig. 3, Table 1).

The article "High Expression of RIOK2 and NOB1 Predict Human Non-small Cell Lung Cancer Outcomes" was retracted in 2023. Reasons: duplicated images; original data or images not available; unreliable results or conclusions; concerns about the data.

In previous studies, we have found an association between high NOB1 expression and NSCLC in 70 patients with NSCLC, and NOB1 expression is related to a poor prognosis in patients with resected NSCLC^12^,^13^. NOB1, which was first isolated by using the yeast two-hybrid screening method^34^, is a nuclear protein that serves as a chaperone for joining the 20S proteasome with the 19S regulatory particle in the nucleus, thereby facilitating the maturation of the 20S proteasome^35^,^36^. Additionally, NOB1 plays a significant role in tumourigenesis and is related to poor prognoses in various cancers^5^. In this study, NOB1 was further studied in 153 patients, and high NOB1 expression was observed in both the NSCLC cell lines and tissues. The results of the IHC analysis of the 153 patients showed that the positive expression of NOB1 was significantly associated with the TNM clinical stage (*P* = 0.003), lymph node metastasis (*P* = 0.017) and differentiation (*P* = 0.030) (Fig. 3, Table 1).

Previous studies have suggested that both RIOK2 and NOB1 are important accessory factors in ribosome assembly^15^,^16^,^17^,^18^,^20^ and that these proteins play a significant role in the progression of the cell cycle. Thus, these proteins are closely related to the proliferation and metastasis of malignant tumours, and they interact with each other^19^,^20^. The results of this study showed that both RIOK2 and NOB1 were significantly upregulated in NSCLC cell lines and tissues. The IHC analysis also indicated that both RIOK2 and NOB1 can be used as prognostic factors for the overall survival rate. Moreover, significantly positive correlations were observed between the expression of RIOK2 and NOB1 in the 153 NSCLC cases (χ^2^ = 0.606, *P* < 0.001) (Fig. 4). The survival analyses showed that patients who presented with high expression levels of both RIOK2 and NOB1 had the lowest overall survival rates.

In summary, this study demonstrates that both RIOK2 and NOB1 play key roles as prognostic markers for poor outcomes in NSCLC patients, and although high expression levels of either RIOK2 or NOB1 were associated with a poor survival rate, the high expression of RIOK2 and NOB1 together resulted in the lowest survival rates. This finding suggests that performing simultaneous detection of RIOK2 and NOB1 expression has the potential to improve the diagnostic rate in early stages of NSCLC. Moreover, RIOK2 and NOB1 might be potential therapeutic targets for NSCLC therapy.

The article "High Expression of RIOK2 and NOB1 Predict Human Non-small Cell Lung Cancer Outcomes" was retracted in 2023. Reasons: duplicated images; original data or images not available; unreliable results or conclusions; concerns about the data.

## Additional Information

**How to cite this article**: Liu, K. *et al*. High Expression of RIOK2 and NOB1 Predict Human Non-small Cell Lung Cancer Outcomes. *Sci. Rep.* **6**, 28666; 10.1038/srep28666 (2016).

## Figures and Tables

**Figure 1:** RIOK2 and NOB1 mRNA expression levels in NSCLC cells. (**a**) The RIOK2 mRNA level in the NSCLC cell lines (A549, H1299, H1975 and H1650) was higher than that in the normal lung cell line (BEAS-2B); (**b**) The NOB1 mRNA level in the NSCLC cell lines (A549, H1299, H1975 and H1650) was higher than that in the normal lung cell line (BEAS-2B).

**Figure 2:** RIOK2 and NOB1 mRNA expression levels in NSCLC tissues compared with normal tissues. (**a**) The mean RIOK2 mRNA expression level was higher in the tumour tissues (2.16 ± 0.57) than in the corresponding paired adjacent normal lung tissues (0.46 ± 0.21) (*P* < 0.001); (**b**) The mean NOB1 mRNA expression level was higher in the tumour tissues (1.06 ± 0.23) than in the corresponding paired adjacent normal lung tissues (0.87 ± 0.16) (*P* = 0.014).

**Figure 3:** Representative patterns of RIOK2 and NOB1 immunohistochemical staining in NSCLC tissues as determined by IHC with TMA sections. (**a**) a weak RIOK2 staining in well-differentiated NSCLC tissues, b positive RIOK2 staining in moderately differentiated NSCLC tissues, c strong positive RIOK2 staining in poorly differentiated NSCLC tissues, d absent RIOK2 staining in an isotype control, e weak NOB1 staining in well-differentiated NSCLC tissue, f positive NOB1 staining in moderately differentiated NSCLC tissue, g strong positive NOB1 staining in poorly differentiated NSCLC tissue, and h absent RIOK2 staining of in an isotype control (200×). (**b**) Protein expression of RIOK2 in the NSCLC patients as detected by western blotting of the fresh frozen tissue samples (T: NSCLC tumour tissue, N: paired adjacent normal lung tissue).

**Figure 4:** Correlation between the expression of RIOK2 and NOB1 in NSCLC tissues.

**Figure 5:** Kaplan-Meier survival curves for the cumulative (cum) overall survival according to the log rank test. (**a**) The overall survival rate of the NSCLC patients with high RIOK2 expression (green line) was significantly lower than that of the patients with low or no expression (blue line). (**b**) The overall survival rate of the NSCLC patients with high NOB1 expression (green line) was significantly lower than that of the patients with low or no expression (blue line). (**c**) The overall survival rate of the NSCLC patients with high RIOK2 and NOB1 expression (green line) was significantly lower than that of the patients with low or no expression or single high RIOK2 or NOB1 expression (blue line).

The article "High Expression of RIOK2 and NOB1 Predict Human Non-small Cell Lung Cancer Outcomes" was retracted in 2023. Reasons: duplicated images; original data or images not available; unreliable results or conclusions; concerns about the data.

**Table 1:** Association of RIOK2 and NOB1 expression with clinicopathological parameters in NSCLC patients.

Clinicopathological parameters	Case No.	RIOK2, n (%)		Pearson *χ*2	*P* value	NOB1, n (%)		Pearson *χ*2	*P* value
		Low or no	High			Low or no	High		
Total	153	83(54.25)	70(45.75)			87(56.86)	66(43.14)		
Gender				0.653	0.419			1.410	0.235
Male	82	42(51.22)	40(48.78)			43(52.44)	39(47.56)		
Female	71	41(57.75)	30(42.25)			44(61.97)	27(38.03)		
Age, yr				3.184	0.074			2.294	0.130
<60	71	44(61.97)	27(38.03)			45(63.38)	26(36.62)		
≥60	82	39(47.56)	43(52.44)			42(51.22)	40(48.78)		
Smoking status				0.914	0.339			1.661	0.197
No	72	42(58.33)	30(41.67)			37(51.38)	35(48.61)		
Yes	81	41(50.62)	40(49.38)			50(61.73)	31(38.27)		
Tumour diameter, cm				2.786	0.095			1.339	0.247
<3	94	56(59.57)	38(40.43)			50(53.19)	44(46.81)		
≥3	59	27(45.76)	32(54.24)			37(62.71)	22(37.29)		
TNM clinical stage				43.778	0.000**			8.610	0.003*
I and II	103	75(72.82)	28(27.18)			67(65.05)	36(34.95)		
III	50	8(16.00)	42(84.00)			20(40.00)	30(60.00)		
Lymph node metastasis				27.222	0.000**			5.666	0.017*
No	63	52(82.54)	13(20.63)			43(68.25)	20(31.75)		
Yes	90	33(36.67)	57(63.33)			44(48.89)	46(51.11)		
Differentiation				6.896	0.018*			5.802	0.030*
Well	2	2(100.00)	0(0.00)			2(100.00)	0(0.00)		
Moderately	99	60(60.61)	39(39.39)			62(62.63)	37(37.37)		
Poorly	52	21(40.38)	31(59.62)			23(44.23)	29(55.77)		

*P < 0.05, **P < 0.001.

**Table 2:** Univariate and multivariate Cox analysis of the overall survival.

Variable	Univariate analysis			Multivariate analysis		
	HR	*P* value	95% CI	HR	*P* value	95% CI
RIOK2						
Low vs. High	2.878	0.000**	1.852–4.474	2.105	0.003*	1.286–3.445
NOB1						
Low vs. High	2.030	0.001*	1.327–3.104	1.858	0.005*	1.207–2.862
Gender						
Male vs. Female	0.715	0.124	0.467–1.096			
Age, yr						
<60 vs. ≥60	1.099	0.662	0.719–1.681			
Smoking status						
No vs. Yes	1.054	0.807	0.691–1.607			
Tumour diameter (cm)						
<3 vs. ≥3	1.641	0.021*	1.078–2.502			
TNM clinical stage						
I and II vs. III	3.381	0.000**	2.191–5.216	2.166	0.002*	1.331–3.524
Lymph node metastasis						
No vs. Yes	1.795	0.010*	1.148–2.806			
Differentiation						
Well vs. Moderately vs. Poorly	2.172	0.000**	1.436–3.286			

HR, hazard ratio; CI, confidence interval. *P < 0.05, **P < 0.001.
